# Application of Accelerometer to Monitor Students' Exercise Load in 50 m Round Trip

**DOI:** 10.1155/2022/3142677

**Published:** 2022-06-29

**Authors:** Hao Li, Meng Xu

**Affiliations:** ^1^Department of Sports Welfare Education, Woosuk University, Jeonju 55338, North Jeolla, Republic of Korea; ^2^Department of Physical Education, Honam University, Gwangju 62397, Metropolitan City, Republic of Korea

## Abstract

With the further advancement of microelectronics innovation and sensors, sensors can be broadly implanted in cell phone gadgets, compact gadgets, and so forth. The utilization of speed increase sensors for human running checking has expansive application possibilities. From one perspective, the everyday development of the human body is firmly connected with the physical and emotional wellness of the person. Observing the day-to-day developments of the human body is of incredible importance in planning a logical running activity plan and working on actual wellbeing. On the other hand, it is also of practical value to monitor human abnormal movements. This kind of abnormal movement caused by accidental falls can bring certain harm to the human body. Real-time monitoring of the fall can provide timely assistance to the person and reduce the risk brought by the fall. This article analyzes and summarizes the research theories and common research methods in the field of 50 m round-trip movement monitoring based on the acceleration sensor. According to the process of 50 m round-trip movement pattern recognition, the data collection, preprocessing, feature extraction, and selection of 50 m round-trip movement are evaluated. The classification and recognition of each module were analyzed. This article proposes a human body motion recognition mechanism based on acceleration sensors by looking at the three trademark upsides, the wavefront edge, wavefront limit, and time stretch between the pinnacle and valley of the speed increase sensor vertical information waveform, and joining the rule of choice tree order to accomplish the activities of hunching down, taking off, and running. To get an accurate recognizable proof and recognize ways of behaving, a human fall identification calculation is proposed. This calculation removes human movement attributes throughout the fall and focuses on four sorts of falls: forward fall, reverse fall, left fall, and right fall by utilizing the connection of the three tomahawks of the speed increase sensor. The trial results show that the normal right acknowledgment pace of the human body's 50 m full-circle running way of behaviour is more than 90%, which has specific useful application esteem.

## 1. Introduction

In recent years, the majority of experts and scholars have explored all aspects of physical education teaching, aware of the importance of the appropriate physiological load borne by students in physical education, and have taken the load standard as an important index to measure the achievement of physical education teaching objectives. With the development of society, the pace of life is accelerated, work efficiency is improved, and leisure time is relatively prolonged. More and more people want to strengthen their physique, adjust their mental state, and enrich cultural life through physical exercise. There are many kinds of day-to-day exercises of the human body, including running, strolling, going all over steps, sitting, standing, and different games. Moreover, the energy utilization relationship compared to these different day-to-day sports is likewise unique, so it is vital to screen and recognize the running heap of the human body in light of the speed increase sensor, which is additionally the primary examination subject of numerous specialists as of now. For example, the pedometer designed by an acceleration sensor can effectively record the walking steps and distance of the human body and calculate the energy consumption of the human body in a period of time using the relationship between human steps and energy consumption, which is of great significance in human health and other aspects of life.

Due to the importance of using acceleration sensors to monitor human movement research, many research teams have begun to study acceleration sensor technology and have achieved good results. For example, Saiki and others put a solitary three-pivot speed increase module at the human wrist position. And utilizing brain fluffy classifiers in a group and recognizing the speed increase signals gathered, the acknowledgment impact is better [1]; Wang et al. utilized a smaller than usual three-pivot speed increase sensor and designed a home checking framework for the older. As a wearable conduct acknowledgment framework, it utilizes multifacet discernment to distinguish nine everyday ways of behaving of the old and can speak with cell phones through the Zigbee convention. The acknowledgment rate and ongoing has a serious level of fit [2]; Tu and others chose to embed a three-axis acceleration sensor in the Philip NWS behavior monitor to collect acceleration information of the human body in various motion states by placing it on the human waist, using Bayesian classifier to identify a variety of sports states including walking, cycling, and driving [3]. Wang led research on the utilization of PDA association through the three-hub speed increase sensor that accompanies the cell phone. He removed an assortment of time-space highlights from the gained speed increase information and utilized a multiclass support vector machine arrangement strategy to complete nine kinds of human body development classification acknowledgment [4].

In the examination of observing the human body's 50 m ever-changing running, it is a decent technique to involve the speed increase sensor for testing. For the model, the Finnish organization has accomplished a progression of exploration results utilizing a solitary speed increase sensor to perceive human movement [5]. A three-axis acceleration sensor is placed on the back of the human body to identify the daily behavior of the human body. At the same time, the human motion consumption is estimated by recording the number of occurrences of the movement. However, accurate motion recognition requires the fusion of multiaxis data, which still brings a higher computing overhead. We collect human body information through a single acceleration, extract human motion characteristics, use the SVM algorithm to classify different actions, and achieve a high recognition rate; and propose a multilayer classifier model based on a neural network; the classification effect is ideal. However, the above methods are relatively complicated, and the system calculation overhead is large.

This article examines and sums up the exploration speculations and regularly involved research strategies in the field of human movement checking in view of speed increase sensors and proposes a human body movement acknowledgment technique in light of a solitary speed increase sensor. It is innovative and experimental. The method combines the decision tree classification algorithm to effectively identify three actions of the human body: running, jumping, and squatting. In view of the investigation and examination of existing fall identification calculations, this article proposes a human fall discovery calculation in light of a three-pivot speed increase sensor. The algorithm proposed in this article can effectively identify fall behavior in different directions while maintaining a high recognition accuracy and also has high real-time performance. The experimental results show that the average correct recognition rate of this article in monitoring the human body's 50 m round-trip running behavior reaches over 90%.

## 2. Proposed Method

### 2.1. Human Motion Monitoring Process

Physical education sports load refers to a series of physiological burdens borne by students' body in physical education. Its load standard is an important index to measure the achievement of physical education teaching objectives. The measurement methods of sports load in physical education can be divided into the direct measurement method and indirect measurement method. The direct measurement method uses a pedometer, accelerometer, heart rate telemetry method, etc., while the indirect measurement methods include the indirect calorimetry method and questionnaire survey method [6]. This article concentrates on the human movement checking in light of speed increase sensors as per the examination thoughts of measurable example acknowledgment. The overall course of factual example acknowledgment comprises information assortment and information preprocessing, include extraction and determination, arrangement, and acknowledgment [7]. The general process of human motion monitoring is shown in Figure 1.

#### 2.1.1. Acceleration Sensor

An acceleration sensor is an electronic device that can measure the acceleration force of an object. Compared with the remote sensing device, it measures its own motion. Its main working principle is as follows: first, convert the acceleration signal measured by the point to be measured into the corresponding electrical signal, which is realized through the sensitive element, then use the signal conditioning circuit in the preamplifier circuit to increase its signal-to-noise ratio, then use the analog-to-digital conversion to convert the analog signal into the corresponding digital signal, and finally send it to the processor and memory for data storage and display [8]. Acceleration sensors can be divided into piezoresistive sensors, piezoelectric sensors, capacitive sensors, servo sensors, and so on. The piezoresistive acceleration sensor mainly uses its own diffusion resistance to measure the acceleration, and different changes output different voltages to reflect the current acceleration [9]. The piezoresistive sensor can directly output voltage signals and does not require complicated circuit interfaces. This is its biggest advantage. The structure of the piezoelectric acceleration sensor is similar to that of the piezoresistive sensor. The difference is that piezoelectric materials such as piezoelectric crystal and piezoelectric ceramics are used to replace piezoresistive materials to induce the change of acceleration; capacitive acceleration sensor is a capacitance sensor based on the capacitance principle. It has the advantages of good sensitivity, good damping characteristics, and small volume. It has been widely used in vehicle system, smartphone platforms, and other fields. Servoacceleration sensor is a closed-loop test system, which has the characteristics of good dynamic performance, large dynamic range, and good linearity. It can be widely used in high-precision inertial navigation and inertial guidance system. Acceleration sensors can be used in the field of human health monitoring and can be used to measure human blood pressure, pulse, heart rate, and other indicators [10]. This human information can provide some help for clinical medical treatment; it can also be used in the field of handheld device context-awareness. It can sense the user's actions through the acceleration sensor and know what the user is doing, what relationship between the user and the handheld device, whether it is in the pocket or in the hand, etc.

#### 2.1.2. Data Collection

To gather human speed increase information, most early scientists planned particular equipment securing hardware. By and large, a framework including a majority of modules like a sensor module, a showcase module, and a remote correspondence module is intended to finish the information assortment work. This strategy for gathering information and examining information requires an individual plan for every module and afterward incorporates it into a framework to finish the information assortment work [11]. As of late, with the advancement of compact cell phones, numerous cell phones have incorporated speed increase sensors, showcases, and correspondence capacities. This sort of savvy cell phone that incorporates speed increase sensors, show screens, and intuitive buttons is regularly involved by analysts in the data procurement stage.

The day-to-day development of the human body is exceptionally confounded and variable. Various activities include various pieces of the body, and the power of the human action is additionally unique. By and large, for various games' ways of behaving, it is important to correspondingly plan the wearing place of the sensor on the human body, and simultaneously, the number of sensors required should be considered. Through the particular thought of the position and number of sensors, it is feasible to take compelling techniques to more precisely recognize different human developments.

The sensors at different positions have different sensitivity to the same kind of motion. At the same time, the acceleration data of the human body collected are very different due to the different positions of the sensors. In addition, because some systems are designed with the user 's wearing comfort and practical value in mind, there are certain restrictions on the location of the sensors. Therefore, when selecting the position of the sensor, it is necessary to consider multiple convenient factors in order to select an appropriate placement solution.

#### 2.1.3. Pretreatment

For the most part, when the speed increase sensor gathers speed increase signals, it additionally contains a few superimposed gravity speed increases and different commotions. Commotion is brought about by human body shake, free or tumbling off of wearable sensor gadgets, and estimation clamor of the actual framework. Preprocessing is generally performed before feature extraction of human motion signals. Signal preprocessing techniques generally include denoising, windowing, and tilt correction.

Because in the process of monitoring and identifying human motion, the collected acceleration data are generally relatively long, it is not suitable to directly perform feature extraction and classification recognition on signals. Therefore, window segmentation of acceleration signals is usually performed [12]. Window division alludes to partitioning the movement signal into many humble fragments, and each time portion is known as a window. The most well-known technique is to utilize a sliding window to separate the sign. The sliding window isolates the movement signal into a few time sections of a similar length. The sliding window is a basic and down-to-earth division technique, which is truly appropriate for frameworks with high ongoing necessities.

Notwithstanding the sliding window division strategy, the ordinarily involved technique for signal division is the occasion-based window. Occasion-based window division alludes to the division of movement signals into portions with various time lengths. Each window represents an event, the start of the window represents the beginning of the event, and the end of the window represents the end of the event [13].

#### 2.1.4. Feature Extraction and Selection

In pattern recognition theory, feature extraction refers to measuring the essential features and attributes of the object to be identified before classification and recognition so as to obtain the pattern describing the object. This process is the process of feature extraction. It can be described as a set of metric values (*x*_1_, *x*_2_,..., *x*_*L*_) to generate new *m* features (*y*_1_, *y*_2_,..., *y*_*m*_) as a dimensionality reduction classification through some transformation hi (·) feature, where *i* = 1,2,…, *m*; *m* < *L*.

Feature selection refers to the selection of features that have a greater effect on classification under certain criteria to complete the task under the premise of meeting a certain correct recognition rate [14]. It can be described as selecting a subset for classification from the *L* metric value sets {*x*_1_, *x*_2_,..., *x*_*L*_} according to certain criteria as the classification feature of the reduced dimension (m dimension, *m* < *L*).

Include extraction and determination rely upon explicit areas, and explicit issues require information direction in the comparing spaces. In down-to-earth applications, some arrangement calculations are not advantageous to characterization with more element values. Now and then, such a large number of highlights will decrease the practicality of the calculation. In order to make the feature better represent the object and facilitate the classification and recognition, the following conditions are usually required when selecting the feature:

1. The amount of effective identification information provided by the feature should be as large as possible. Such features have good separability and are convenient for the classifier to classify better.
2. Try not to select those features that are ambiguous and difficult to distinguish easily.
3. Choose only one of the repeated and highly relevant features because strong correlation does not add more classification information, and they are also essentially duplicates, which is not necessary.
4. The quantity is as small as possible and the data are easy to obtain, so the loss of information amount will also be reduced.
5. It is convenient and economical to extract features, which is convenient for practical operation.

In the field of human movement acknowledgment, include extraction is a significant piece of the whole acknowledgment process. The speed increase signal waveform cannot be straightforwardly perceived by the classifier, nor would it be able to be utilized to address human movement qualities actually [15]. Thus, we really want to perform highlight extraction on the speed increase signal, remove helpful data as element values, and afterward consolidate the classifier calculation to perceive human movement. As of now, include extraction strategies regularly utilized in the field of human movement acknowledgment can be partitioned into time-space highlight extraction, recurrence area include extraction, wavelet extraction, etc.

Time-space highlights: also called measurable elements of signs, include extraction is performed utilizing probabilistic strategies [16]. Vector highlights are straightforwardly extricated from the time waveform of speed increase. Time-space highlights are the most generally involved technique in the human movement acknowledgment process, on the grounds that the time area include extraction strategy is moderately straightforward and how much estimation is not huge. Regularly utilized time-space highlights are mean, change, energy, time area reconciliation, etc. Many time-space highlights have explicit actual implications. For instance, the mean worth can be utilized to address the DC part of a sign, and the difference can be utilized to depict the steadiness of a speed increase signal.

Frequency domain feature: it is a feature that reflects the motion signal from the perspective of the frequency domain. The most common method for converting the time domain to the frequency domain is the fast Fourier transform. Some researchers use the absolute value of the FFT coefficients of human motion signals in a window as the characteristic values. Some people also add the sum of the FFT coefficients as the energy of the motion signal to the feature vector [17–19]. Because the frequency domain features are generally based on FFT, and the fast Fourier transform calculations are generally large, the frequency of using the frequency domain features is not as high as the time domain features.

Wavelet include: it is a technique that joins time area data and recurrence space data. The wavelet examination strategy primarily utilizes a bunch of wavelet reference capacities to change over movement signals into itemized flags and surmised signals with various perception exactness. It can simultaneously describe the time domain characteristics and frequency domain characteristics of signals [20, 21]. Some existing studies use the wavelet transform technology to extract human motion signal features.

#### 2.1.5. Classification and Recognition

The recognition methods used in human motion recognition based on acceleration sensor generally belong to statistical pattern recognition. After the feature vector is obtained by feature selection and extraction, it is necessary to select an appropriate classification method to classify the recognized objects according to the known feature vector. The choice of classification method plays an important role in the entire recognition system [22]. There are numerous strategies to tackle the order issue. The order strategies that are regularly utilized are choice trees, Naive Bayes, K-closest neighbors, support vector machines, fake brain organizations, etc.

*(1) Decision Tree*. Decision tree is one of the main technologies for classification and prediction. Decision tree learning is a case-based inductive learning algorithm. It focuses on inferring the classification rules represented by a decision tree from a group of unordered and irregular cases [23]. The decision tree selecting the optimal test attributes at each node is the key to the decision tree algorithm. A commonly used method is to use the information gain entropy to calculate the required test attributes. Suppose *S* represents a set of *s* training samples, and there are *m* classes *C*_1_,…, *C*_*m*_ [24], where *S*_*i*_ is the number of samples in *C*_*i*_, and the probability that the sample belongs to *C*_*i*_ is represented by *p*_*i*_. *s*/*s*_*i*_ is used to estimate the information entropy of a given sample set as follows:

(1) $$\begin{array}{c} I\left(s_{1},\ldots ,s_{m}\right)=-\sum_{i=1}^{m}p_{i}\log_{2}\left(p_{i}\right). \end{array}$$

It can be seen from formula (1) that if it is assumed that attribute A is selected as the test attribute, the sample set *S* can be divided into *v* subsets {*S*_1_,…, *S*_*m*_}, and let *s*_*ij*_ be the number of *C*_*j*_ samples in the subset *S*_*j*_, then it is divided by the test attribute A. The information entropy of the subset can be expressed as follows:

(2) $$\begin{array}{c} E\left(A\right)=\sum_{i=1}^{v}\left(s_{ij}+\cdots +s_{ij}/s\right)I\left(s_{ij},\ldots ,s_{ij}\right). \end{array}$$

Among them,

(3) $$\begin{array}{c} I\left(s_{ij},\ldots ,s_{ij}\right)=-\sum_{i=1}^{m}p_{ij}\log_{2}\left(p_{ij}\right). \end{array}$$

Here, *p*_*ij*_=(*s*_*ij*_/|*s*_*j*_|) is mainly used to estimate the probability that each type of sample in *S*_*j*_ belongs to *C*_*i*_.

The samples of each category can be well divided, and the corresponding information entropy will also become smaller so that the overall information entropy will become smaller.

Finally, by comparing the difference between *E* (*A*) and *I*(*s*_1_,…, *s*_*m*_), the information gain entropy of the selected test attribute A can be obtained, and so on, the attributes B and C can be calculated. Obviously, when the information gain entropy get larger, this means that using this attribute as the splitting attribute can distinguish different samples well [25]. The process of the decision tree algorithm is shown in Figure 2.

*(2) Naive Bayes*. A Bayesian classification algorithm is an algorithm that uses statistical probability theory to classify, such as a naive Bayesian algorithm. Its basic idea is to use the Bayesian theorem to calculate the probability that a sample to be classified belongs to a certain category, compare the calculated probability, and select the category with the largest probability as the category of the sample. The establishment of Bayes' theorem needs to meet certain prerequisites, that is, the premise of condition independence, but this premise cannot be generally satisfied in practice, which will reduce the accuracy of this classification method.

Bayes' theorem is shown in the following formula:

(4) $$\begin{array}{c} P\left(C_{i}|X\right)=\frac{P\left(X|C_{i}\right)P\left(C_{i}\right)}{P\left(X\right)}, \end{array}$$

where *P*(*C*_*i*_*|X*) represents the probability that *X* belongs to the category *C*_*i*_. Because the distribution function *P*(*X*) is the same for different samples *X*, only the size of *P*(*X|C*_*i*_)*P*(*C*_*i*_)*|* needs to be calculated. *P*(*C*_*i*_) can be estimated from the number of samples in the training set. When calculating the conditional density probability *P*(*X|C*_*i*_), for simplicity, it is generally considered to be independent for different classes, and the likelihood function derived from it is as follows:

(5) $$\begin{array}{c} P\left(X|C_{i}\right)=\prod_{k=1}^{n}P\left(x_{k}|C_{i}\right). \end{array}$$

Among them, *x*_*k*_ represents the components of the n-dimensional feature vector *X*.

For discrete feature attributes, conditional probability can be estimated by calculating the number of attribute values *x*_*k*_ in *C*_*i*_, while there are continuous attributes.

The conditional probability density should be estimated statistically [26].  Figure 3 is the flowchart of the Bayesian algorithm.

### 2.2. Human Motion Monitoring

Normal strategies for recognizing human developments incorporate nonspeed increase sensor acknowledgment techniques like video, picture investigation, and sound examination. Among them, the human movement acknowledgment strategy in light of video and picture investigation has a greater expense, higher necessities on the climate, and unfortunate adaptability and can be perceived in unambiguous regions.

#### 2.2.1. Data Preprocessing

*(1) Acceleration Sensor Placement*. The acceleration data obtained by placing the sensor on the chest position are relatively stable, the sensitivity is moderate, and it is also convenient for people to carry (you can put the device with the sensor in the jacket pocket) [27]. In this article, the study of human motion monitoring mainly considers the stability of the acceleration data and the performance suitable for carrying. Therefore, the front chest position is selected to place sensors to study human motion.

A three-hub speed increase sensor is put on the facade of the human body. The three tomahawks of the speed increase sensor are X-hub, Y-hub, and Z-hub. The Y-hub corresponds to the upward course of the human body and the positive pivot focuses on the upper part. In the forward bearing, the *X* pivot is opposite to the plane made out of Y and Z, as shown in Figure 4.

*(2) Vertical Correction*. During the development of an individual, in the event that the sensor is not totally fixed on the human body, the place of the sensor might change, and the results of the three tomahawks of speed increase cannot precisely mirror what is happening in the human body. On the off chance that the sensor is totally fixed to the human body, it will truly influence the wearing solace, which will diminish the viable worth of this exploration. To diminish the mistake brought about by the difference in the sensor position, this article utilizes the upward adjustment technique for the speed increase sign to concentrate on human movement. Since the speed increase information in the upward bearing (inverse to gravity) gives more significant trademark data in human development, this part principally utilizes the upward course to concentrate on human development.

On the ground, the gravity component of the acceleration sensor is always constant; that is, it always points vertically downwards on the ground. Therefore, when the acceleration sensor is stationary, the vector sum of its three axes is equal to the acceleration *g* of gravity. The vector synthesis is shown in Figure 5.

(6) $$\begin{array}{c} g=\left(a_{x},a_{y},a_{z}\right). \end{array}$$

When the human body moves, the values of the three axes of the acceleration sensor represent the sum of the acceleration component and the gravity component generated by the human body on each axis. The gravity component does not affect our research, so the vertical component in this article includes the gravity component and the human acceleration component.

#### 2.2.2. Selection of Human Motion Characteristic Values

In this article, in the selection of human motion feature values, we mainly consider selecting the feature values that are most effective for motion classification and using as few feature values as possible to complete the same classification, so as to reduce the computational complexity. In this article, three characteristic values of the wavefront threshold, wavefront threshold, and peak-to-valley time interval are extracted from the time domain of the acceleration signal to realize the effective recognition of the three movements of running, taking off, and squatting in human daily activities.

*(1) Prepeak Threshold*. During the development of the human body, the upward sign of speed increase will constantly change. The most extreme worth of the sign throughout some stretch of time is the wave peak. The wave peak can all the more likely mirror the power of the human body's development—the pinnacle worth of the wave is bigger. Since the recurrence of various activities of the human body is unique, the force of the activity is additionally unique, so the pinnacles created by various activities will likewise be unique. This article chooses a threshold value before the peak of the acceleration signal as the eigenvalue, which has obvious effects on the recognition of the three movements of running, jumping, and squatting.

*(2) Threshold before Trough*. As opposed to the wave top, the base worth of the sign throughout some undefined time frame is the wave box. The box can all the more likely mirror the power of the descending development of the human body. The bigger the prompt box esteem, the more prominent the adjustment of the stance of the human body. We pick an edge before the box shows up as another eigenvalue.

*(3) Peak and Valley Time Interval*. Top-to-valley time stretch alludes to the time distinction between two contiguous pinnacles and valleys. Because of the different cycle frequencies of various activities, the time span between the event of pinnacles and valleys is unique. The time stretch among pinnacles and valleys can mirror the human body. The recurrence of intermittent movement is additionally a significant element esteem in recognizing human developments in this review.

## 3. Experiments

### 3.1. Experimental Platform

The human motion recognition method proposed in this article has been verified on smart terminals. The smart terminal uses the Android operating system and is equipped with a LIS3DH acceleration sensor. LIS3DH is a three-axis digital acceleration sensor from STMicroelectronics. It is packaged in a 16-pin plastic package and has a small and slim profile with a size of only 3 mm × 3 mm × 1 mm. It adopts digital output, which avoids the use of other chips for analog-to-digital conversion. The acceleration sensor LIS3DH has *X*, *Y*, and *Z* acceleration outputs with three degrees of freedom. It can sense the movement information of the human body in all directions. The measuring range is within ±2 g/± 4 g/± 8 g/± 16 g, and the working current consumption is at least 2 *μ*A. LIS3DH can provide very accurate measurement data output and can still maintain excellent stability under rated temperature and long-term work. The sampling rate of the sensor is adjustable between 1 and 5000 Hz. The sampling frequency set in this article is 50 Hz, and 50 samples are collected per second. A low sampling rate can not only reduce system power consumption but also reduce noise interference.

### 3.2. Experimental Collection

There were 12 participants, including 5 females and 7 males, aged 23–27 years, height 156 cm–180 cm, weight 48 kg–75 kg. The mobile terminal equipped with the LIS3DH acceleration sensor was placed in the pocket of the experimenter's chest shirt, and the experimental location was selected in the open air. Each experimenter made three movements of running, taking off, and squatting 10 times, and the interval between the movements was more than 20 s so that the experimenters could adjust themselves to the normal state. Among them, take-off and squat are both in situ actions. The experimenter performs tests according to his normal state. We have no specific restrictions on the actions performed by the experimenter. We test in accordance with our usual state. The experimenter is required to run more than 5 steps and test according to his normal running state.

### 3.3. Experimental Methods

Before the first experimental test, the basic information of the subject is measured and recorded. Record height, weight, age, body composition, etc. Wear the LIS3DH acceleration sensor before each exercise. Second, the subject took a sitting position, and after sitting for 10 minutes before exercise, the blood pressure and heart rate were measured twice with an electronic sphygmomanometer, and the average of the two measured values was the quiet blood pressure and the quiet heart rate. Third, each exercise is performed in accordance with the load intensity from small to large, and the subject is fully rested (sitting for 10 minutes before exercise and resting after each load). Achieve the quiet heart rate and perform the lower load standard: no more than 3 times (including 3 times) the quiet heart rate before the upper load exercise. The subject stood up from the sitting position, walked to the running platform, turned on the running platform, gradually accelerated to the target speed, and after moving for 3 minutes at the target speed, gradually decreased to a speed of 0.8 km/*h*. Go to the sitting position and take a rest. Record the subjective physical feeling, running distance, and running time immediately after exercise. After a full rest (approximately 15–30 minutes after the end of the exercise), the average heart rate returning to no more than 3 times is considered to return to a quiet level. Record the rest time, approximately determine how long it takes to recover to a quiet heart rate, and ensure that the second and third rest periods are basically the same for the formal experiment. Fourth, measure blood pressure and heart rate, determine that it has reached a quiet level, and perform the next load. The quiet heart rate is the same as above. Record your heart rate throughout the process with a Finnish POLAR telemeter computer. Fourth, after 48 hours, the same exercise regimen as the previous time was used. Participants were required to use the same time and clothing as the last test for the second exercise.

## 4. Discussion

### 4.1. Analysis of Antifall Detection of Human Body 50 m Round-Trip Running Based on Acceleration Sensor

The trial results recorded the right recognizable proof, oversight, and misleading upsides of falls. Among them, right recognizable proof demonstrates the right ID of the fall and its heading; underreporting indicates that the experimenter did not recognize the fall behavior after falling in a 50 m round trip; and false alarms indicate that after the experimenter falls in a certain direction, the system judges it as fall in other directions. We made a point-by-point record of the whole trial process, and the trial factual outcomes are displayed in Table 1.

From Table 1, it can be seen that the algorithm proposed in this paper has a correct recognition rate of more than 90% of the fall behavior, and there are no false positives in the entire experimental process. The recognition rate of falls in each direction is different. The recognition rate of falls before a round trip to 50 m is low, and the recognition rates of falls in the other three directions are high. Because the fall experiment in this article is performed consciously, the psychology of the experimenter will have an impact on the experimental results.

During the 50 m round-trip forward fall, the experimenter's simulation of the real fall is not enough, so sometimes, the threshold set by the algorithm is not reached, which will cause false negatives. After analyzing the experimental results, it is found that the fall recognition rate of males in this article is significantly higher than that of females. This is because male experimenters have stronger psychological conditions than females, and the fall speed and amplitude of 50 m round-trip exercise are larger, and the experiment is closer to the real situation. The experiment is shown in Figure 4.

As shown in Figure 6, considering that the human body is generally in a horizontal state after a fall of 50 m of back-and-forth movement, this article calculates the average of the falling direction within the time *T* after the starting point of rest to identify the falling in each direction. This article takes time *T* = 1 s; that is, there are 50 sampling points in the dumping direction axis, and the average value of the sampling points, *M* (az) or *M* (ax), is calculated. According to the range of the dumping direction axis average value, it can be determined in various fall situations.

### 4.2. Comparative Analysis of Attention Quality before and after 50 m Round Trip

In running sports, training athletes' concentration is actually a contradictory effort. Because on the playing field, the factors that affect the athlete 's attention are objective. At this time, when the athlete pays attention to a certain thing, the mental energy consumed is very large, so the athlete 's mental and spiritual feelings are very tired. This causes the athletes to relax mentally and slow their physical activity. In fact, during the 50 m round-trip competition, the athlete insisted on reminding himself to concentrate all the time so that the athlete could not concentrate. The experimental results are shown in Table 2.

As shown in Table 2, by comparing the athletes 'attention quality indicators before and after the 50 m round-trip exercise test, the attention distribution indicators before and after the high-intensity exercise load were significantly reduced (*p* < 0.05), and the athletes' attention span indicators were significantly decreased (*p* < 0.05). The stability index was significantly improved (*p* < 0.05). Note that the transfer index was significantly improved (*p* < 0.05).

Next, this article records the test data of the testers during the 50 m round-trip (a total of 100 m) from 0, 25, 50, 70, and 100 m. “Before” and “after” in the analysis results, respectively, represent before and after exercise. Distribution, stability, concentration, and transfer represent the four qualities of attention: distribution, stability, concentration, and transfer. The experimental results are shown in Figure 7.

As shown in Figure 7, when analyzing the above data, one point needs attention. Although an individual may experience abnormal behavior due to a drop in attention quality level after being subjected to a 50 m round-trip exercise load, the cause is often not caused by a drop in attention quality. We can give an example to illustrate the above two points. In the confrontational ball game, after bearing the load, the athlete cannot quickly shift the focus of attention. After the focus shifts, the attention resources cannot be allocated quickly, resulting in a mistake. The cause of the mistake is not only the result of the athletes' attention to the decline in the distribution speed but also the result of the decrease in the transfer speed. Therefore, when exercising, the abnormal behavior caused by the decline in the quality of the idea is caused by more than two types of attention.

### 4.3. Experimental Analysis of the Recovery of the Load Exercise between the Front and Back 50 m Rounds

After each 50 m round-trip load exercise, the subjects were fully rested. Before the exercise, the quiet heart rate was measured. The measurement standard was to measure the heart rate twice in succession, and the average value was taken as the quiet heart rate. When the heart rate reaches no more than 3 beats per minute compared with the last resting heart rate, it is regarded as the quiet heart rate and the next load is performed. Record the rest time to ensure that the rest time for the 2nd and 3rd exercise is basically the same. The results of the resting heart rate before the load of two or three times of exercise for a group of subjects are shown in Figure 8.

As shown in Figure 8, there was a significant difference in the resting heart rate between the second exercise and the third exercise before the third exercise; that is, there was a difference in the heart rate recovery between the two exercises. In the following analysis, the third test was excluded. In this way, the subject's heart rate can be restored to a quiet state, so that the front and back exercises are consistent.

### 4.4. Analysis of Blood Pressure Recovery before and after 50 m Round-Trip Exercise

Quiet blood pressure measurement before exercise: let the subject sit still for 10 minutes, expose the upper arm, fasten the cuff so that the position of the cuff is equal to the subject's heart, test according to the standard test method, and take the average of two measurements to be quiet blood pressure. Take a full rest after exercise, and measure blood pressure while measuring the quiet heart rate. The test method is the same as above. The results of a group of silent systolic blood pressure tests are shown in Table 3.

As shown in Table 3, the highest systolic blood pressure was 134 mm/Hg and the lowest systolic blood pressure was 117 mm/Hg in the load group. Due to the large individual differences, differences between the highest and lowest systolic blood pressure are observed: 17 mm/Hg. Normal systolic blood pressure was below 140 mm/Hg, and 7 of the 10 subjects had an average quiet systolic blood pressure greater than 120 mm/Hg. In the 50 m reciprocating running load exercise test, the systolic blood pressure before the 50 m reciprocating running load exercise was about 17.33 kPa, about 130 mm/Hg, which means that the subjects showed a quiet systolic pressure higher than normal. This result may be due to the subject's normal physiological response due to imminent exercise, that is, the feedforward phenomenon. Pregnant women also easily cause blood pressure to rise before giving birth, which is mainly caused by active sympathetic nerve transitions, which is also a kind of feedforward phenomenon. Subject No. 9 in the first load group did not meet the requirements because of significant differences in the systolic blood pressure during the second and third times of exercise. All the data of Subject No. 9 were excluded in the following analysis.

The method for measuring the systolic blood pressure of the second group of subjects in the 50 m round-trip running exercise is the same as above.

As displayed in Figure 9, the greatest systolic pulse is 132 mm/Hg, the base systolic circulatory strain is 114 mm/Hg, and the distinction between the most extreme and least systolic circulatory strain is 18 mm/Hg in the two gatherings of 50 m full circle running. There were no massive contrasts in the systolic pulse of the second gathering of subjects during the 50 m full circle pursuing activity previously and the matched *t*-test.

## 5. Conclusions

In this article, the investigation of the human body's 50 m full circle running burden observing in view of speed increase sensors has a place in the field of example acknowledgment, and there are many examination strategies in this field. The examination strategies in light of speed increase sensors can fundamentally be summed up into two classifications: research in view of the combination of different sensors and exploration in view of a single speed increase sensor. Among them, the multisensor-based research technique has a high acknowledgment precision in the acknowledgment of human movement conduct because of the combination of different sensor information; however, then again, the combination of multisensors likewise brings specific computational upward. With the promotion of different portable terminal gadgets, the utilization of a solitary speed increase sensor is becoming more and more extensive, and the pragmatic appropriateness is becoming more and more grounded.

The research in this article uses a single acceleration sensor to extract human features during the 50 m round-trip running load exercise and combines a decision tree classification method to realize a human body's daily motion recognition scheme, which can perform three actions of running, jumping, and squatting. Effective identification: in the study of human abnormal motion, a human fall detection algorithm was proposed. By working out the greatness and difference of the joined speed increase SA and the computation of every hub of the speed increase, it can really recognize falls this way and that of the human body.

In this article, through the correlation analysis of the heart rate index of the 50 m round-trip running test subjects, the stability of the heart rate integral is the highest, the average heart rate and the highest heart rate stability are the second, and the heart rate stability is slightly worse immediately after the exercise and the subjective physical strength. The stability of feeling is the worst, and the stronger the athletic ability, the better the stability of subjective physical feeling.

## Figures and Tables

**Figure 1:** Research process based on statistical pattern recognition.

**Figure 2:** Decision tree algorithm.

**Figure 3:** Bayesian algorithm flowchart.

**Figure 4:** Three-dimensional space coordinates of human acceleration.

**Figure 5:** Three-axis synthesis of the acceleration sensor at rest.

**Figure 6:** Results of different types of falls.

**Figure 7:** Analysis of various attention quality tests before and after loading.

**Figure 8:** A graph of resting heart rate results for a group of subjects.

**Figure 9:** Results of subjects' quiet diastolic blood pressure (*n* = 5, unit: mm/Hg).

**Table 1:** Results of different types of falls.

Action	Total number of experiments	Number of correct identifications	Correct rate (%)	Underreports (%)
Fall forward	24	20	83.33	0

Fall backward	24	22	91.67	0

Fall to the left	24	23	95.83	0

Fall right	24	22	91.67	0

Total	24	87	90.63	0

**Table 2:** Comparison of psychological quality of athletes before and after the experiment.

		N	Before	After	*t*	*p*
50 m before and after exercise	Pay attention to allocation	12	20.24 ± 2.14	18.61 ± 2.01	1.581	<0.05
	Attention span	12	102.14 ± 10.21	100.24 ± 9.45	1.921	<0.05
	Pay attention to stability	12	15.42 ± 2.04	17.32 ± 2.64	2.037	<0.05
	Attention shift	12	104.32 ± 8.01	106.27 ± 8.24	2.107	<0.05

**Table 3:** Quiet systolic blood pressure table of the subjects in the load group (*n* = 5, unit: mm/Hg).

Load subject	Quiet systolic pressure for the second 50-meter round trip	Load subject	The third 50-meter round-trip quiet systolic pressure
1	117.24 ± 3.24	6	119.17 ± 4.52
2	119.20 ± 5.27	7	123.67 ± 4.38
3	132.68 ± 8.61	8	127.44 ± 5.84
4	130.77 ± 4.54	9	125.31 ± 9.47
5	134.26 ± 6.68	10	126.24 ± 3.21

## Data Availability

The data that support the findings of this study are available from the corresponding author upon reasonable request.
